# Clinical Efficacy of PEG-IFN*α*-2a and PEG-IFN*α*-2b in the Treatment of Hepatitis B e Antigen-Positive Hepatitis B and Their Value in Improving Inflammatory Factors and Hemodynamics in Patients: A Comparative Study

**DOI:** 10.1155/2022/3185320

**Published:** 2022-06-11

**Authors:** Nina Jia, Wei Gao, Xiaohong Fan, Hong Gao, Xueqing Li, Biantao Mi, Jie Yang

**Affiliations:** Department of Gastroenterology, The Second Hospital of Shanxi Medical University, Taiyuan, 030001 Shanxi, China

## Abstract

**Objective:**

To compare the merits and demerits of PEG-IFN*α*-2a and PEG-IFN*α*-2b for the treatment of hepatitis B e antigen (HBeAg)-positive chronic hepatitis B (CHB).

**Methods:**

Clinical files from eighty-four CHB patients admitted to the Second Hospital of Shanxi Medical University between January 2018 and January 2019 were retrospectively analyzed and assigned to two groups: group 2a treated with PEG-IFN*α*-2a and group 2b treated with PEG-IFN*α*-2b. The clinical efficacy was compared between the above two arms, and the liver function (ALT, AST, HA, LN, and IV-C), HBV-DNA, HBsAg, HBeAg, and inflammatory factors (IFs, IL-1*β*, IL-6, IL-8, and TNF-*α*) were tested at 12 weeks (T1), 24 weeks (T2), and 48 weeks (T3). The alterations of hemodynamics (SBP, DBP, MAP, and CVP), cardiac function (LVEF and BNP), and the incidence of adverse reactions (ARs) during treatment were recorded. Finally, the patients were followed up for 2 years to investigate the quality of life (QOL) as well as the positive seroconversion rate of HBsAg and HBeAg.

**Results:**

The overall response rate was similar in the two arms (*P* > 0.05). After treatment, the liver function, HBV-DNA, HBsAg, HBeAg, IFs, hemodynamics, and cardiac function were enormously improved (*P* < 0.05), with faster improvement in group 2b compared with group 2a (*P* < 0.05). The investigation of ARs identified notably lower incidence rates of alopecia, thrombocytopenia, and granulocytopenia in group 2a as compared to group 2b (*P* < 0.05). The prognostic follow-up results revealed no distinct difference in the QOL score and the positive seroconversion rate of HBsAg and HBeAg (*P* > 0.05); however, the quantitative results of HBV-DNA, HBsAg, and HBeAg in group 2b were lower than those in group 2a (*P* < 0.05).

**Conclusions:**

Both PEG-IFN*α*-2a and PEG-IFN*α*-2b have excellent and stable therapeutic effects on HBeAg-positive CHB, among which PEG-IFN*α*-2b renders a faster treatment process but higher side effects, which can provide valuable references when choosing a treatment plan for CHB.

## 1. Introduction

Chronic hepatitis B (CHB), one of the most pervasive infectious diseases globally, is caused by hepatitis B virus (HBV) and is highly contagious [1]. As indicated by statistics, the number of known CHB patients worldwide continues to increase, with more than 260 million cases as of 2016 [2]. The incidence of CHB also varies greatly among different regions. In China, India, and other regions with large population density and base, the infection rate has increased significantly [3]. For example, there are over 70 million cases of HBV infection in China, of which more than 40% were finally diagnosed as CHB [4]. At the early stage, CHB presents no other special clinical symptoms except dizziness and anorexia, which are often ignored by patients [5]. However, when there are obvious symptoms, the disease has usually progressed into the middle and late stage when pathological conditions such as liver fibrosis, liver dysfunction, failure, and even liver cancer may occur in patients [6]. On average, approximately 800,000 to 900,000 patients die each year from CHB, a two-to-fourfold increase in mortality compared to 2006, according to the study [7].

Currently, CHB treatment depends largely on conservative therapy, mainly through antivirus, immunomodulation, anti-inflammatory, and liver protection methods to inhibit or eliminate HBV infection in the long term. Among them, nucleoside (acid) analogues and interferon (IFN) are all clinical treatments for CB. Nucleoside (acid) analogues have excellent antiviral effect and good tolerance, but the treatment time is extremely long; Moreover, nucleoside (acid) analogues under selective pressure may cause virus variability resistance, resulting in virologic rebound and liver metabolic disturbance [8, 9]. IFN, on the other hand, plays an anti-HBV effect through the dual effects of HBV replication and immune regulation, with higher serological response and longer sustained virologic response, which is mainly related to molecular pathways. It has the same anti-HBV ability as nucleoside (acid) but faster antiviral effect, so it has been increasingly applied in CHB treatment in recent years [10, 11].

Currently, PEG-IFN*α*-2A and PEG-IFN*α*-2b are commonly used in clinical practice, both of which have well-documented therapeutic effects on CHB [12, 13]. However, the difference between the two types of IFN genes on CHB is still under debate, and there is no authoritative research that indicates which type is more suitable for CHB treatment. Furthermore, we found that previous studies on PEG-IFN*α*-2a and PEG-IFN*α*-2b in treating CHB mostly focused on patients' hepatitis virus infection, ignoring the changes of other vital signs [14, 15]. As we all know, pathological changes such as inflammatory factors (IFs) and hemodynamics are also important links in the occurrence of CHB, which are closely related to the pathology of infection. Thus, the motivation and novelty of this study are to compare the effect of PEG-IFN*α*-2a and PEG-IFN*α*-2b in treating CHB on the change of inflammatory factors and hemodynamics in patients, hopefully, to provide strong evidence for the treatment protocol of CHB.

With the increasing incidence of CHB and its major threat, it is necessary to find a suitable treatment for CHB as soon as possible. This study, undoubtedly, will provide more reliable and comprehensive experimental guidance for future treatment of CHB by investigating the impacts of PEG-IFN*α*-2a and PEG-IFN*α*-2b on clinical efficacy as well as the hemodynamics and IFs of patients with HBeAg-positive CHB.

## 2. Materials and Methods

### 2.1. Patient Data

The study population comprised 84 CHB patients admitted to the Second Hospital of Shanxi Medical University between January 2018 and January 2019. There were 49 males and 35 females, and the mean age was (47.6 ± 7.4) years (range: 34-61). Ethical approval has been obtained for this study, all subjects were aware of the study and signed informed consent. The enrolled CHB patients were assigned to group 2b and group 2a according to treatment plan, with 42 cases in each group.

### 2.2. Eligibility Criteria

Inclusion criteria: (1) presence of clinical manifestations of CHB (constitutional symptoms, anorexia, nausea, jaundice, and right upper quadrant discomfort), together with the confirmed diagnosis of HBeAg-positive CHB after second liver two half-and-half test in our hospital [16]; (2) >18 years old; (3) no liver cirrhosis; (4) complete case data; (5) willingness to participate in this study. Exclusion criteria: (1) hepatitis A, hepatitis C, or reinfection with other hepatitis viruses; (2) autoimmune liver diseases; (3) other cardiovascular and cerebrovascular diseases and hematopoietic system diseases; (4) neoplastic diseases; (5) drug-induced liver injury and alcoholic liver injury; (6) drug allergies; (7) pregnant and lactating women; (8) mental disorders; (9) referrals.

### 2.3. Treatment Methods

After admission, patients in both arms received routine examinations such as second liver two half-and-half and were treated accordingly. Group 2a: 180 *μ*g PEG-IFN*α*-2a (Shanghai Roche Pharmaceutical Ltd., SFDA Approval No. J20070055) was injected subcutaneously once a week. Group 2b: 180 *μ*g PEG-IFN*α*-2b (Xiamen Amoytop Biotech Co., Ltd., SFDA Approval No. S20174005) was injected subcutaneously weekly. Both arms were treated continuously for 48 weeks.

### 2.4. Blood Sample Collection

At 12 weeks (T1), 24 weeks (T2), and 48 weeks (T3) after treatment, 5 mL of fasting venous blood was extracted from patients into coagulation-promoting tubes, which were left at room temperature for 30 min and then centrifuged (1505 × g, 4°C) to obtain serum to be refrigerated at -80°C.

### 2.5. Observational Indicators

#### 2.5.1. Clinical Efficacy

Markedly effective was considered if the symptoms disappeared, the liver function recovered more than 50%, and the liver fibrosis indexes recovered to normal levels. Effective was translated in basically disappeared symptoms and a 10-50% recovery of the liver function. Failure to meet the above standards was considered ineffective. Total effective rate = (markedly effective + effective) cases/total cases × 100%.

#### 2.5.2. Liver Function

The contents of alanine aminotransferase (ALT) and aspartate aminotransferase (AST) were measured using an automatic biochemical analyzer (Sysmex Corporation, Kobe, Japan). (2) The determination of liver fibrosis indexes including hyaluronidase (HA), laminin (LN), type IV collagen (IV-C), and B-type natriuretic peptide (BNP) contents was realized by chemiluminescence. ALT, AST, HA, LN, and IV-C of patients in both arms were recorded at 12 T1, T2, and T3.

#### 2.5.3. Marker Conversion

The detection of serum hepatitis B virus deoxyribonucleic acid (HBV DNA) employed PCR. ELISA was used for determining the expression of hepatitis B surface antigen (HBsAg) and hepatitis B e antigen (HBeAg). HBV-DNA, HBsAg, and HBeAg levels were quantified, and HBV-DNA (HBV − DNA quantification < 2.5lg copies/mL is judged as HBV-DNA negative conversion), HBsAg, and HBeAg negative conversion ratios were calculated.

#### 2.5.4. IFs

ELISA was used for determining the expression of hepatitis B surface antigen (HBsAg), hepatitis B e antigen (HBeAg), as well as IFs IL-1*β*, IL-6, IL-8, and TNF-*α*. The kits were supplied by Shanghai Enzyme Research Biotechnology Co., Ltd., and the operation procedure was carried out strictly in accordance with the instructions.

#### 2.5.5. Hemodynamics and Cardiac Function

The left ventricular ejection fraction (LVEF) was measured by echocardiography. The left femoral artery was continuously monitored for mean arterial pressure (MAP), central venous pressure (CVP), systolic blood pressure (SBP), and diastolic blood pressure (DBP).

#### 2.5.6. Safety

The incidence of adverse reactions (ARs) from admission to discharge was calculated. (8) Prognosis: the prognostic QOL score and positive seroconversion rate of HBsAg and HBeAg (the number of patients with positive HBsAg and HBeAg reexamination results) were recorded.

### 2.6. Follow-Up for Prognosis

Patients in both arms were followed up for 2 years via regular hospital reexamination. The 36-Item Short-Form Health Survey (SF-36) [17] was used to investigate patients' social functioning, role emotional, mental health, and vitality at the end of the 2-year follow-up. Each dimension has a maximum score of 100, and a higher score indicates a better quality of life (QOL). In addition, patients were regularly reviewed for second liver two half-and-half.

### 2.7. Statistical Processing

The statistical method applied in this study was SPSS24.0. The enumeration data was recorded as [*n*(%)], and Chi-square test was used for comparison between groups. The measurement data were recorded in (^−^*χ* ± s); independent samples *t*-test and paired *t*-test were used for comparison among groups, and one-way analysis of variance and LSD post hoc test was used for comparison among multiple groups. A *P* value less than 0.05 was considered to be of statistical significance.

## 3. Results

### 3.1. Comparison of Clinical Baseline Data

In order to ensure the accuracy of the experimental results, we made a statistical comparison of the clinical baseline data of the two groups. The results identified no distinct difference in baseline data such as age and gender between the two arms (*P* > 0.05), suggesting comparability Table 1.

### 3.2. Comparison of Clinical Efficacy

Total effective rate was not statistically different between group 2b (83.33%) and group 2a (90.48%) (*P* > 0.05) Table 2.

### 3.3. Liver Function Comparison

T2 and T3 had witnessed no statistical difference in ALT, AST, HA, LN, and IV-C between the two arms (*P* > 0.05). Whereas, at T1, the above liver function indexes were all lower in group 2b than in group 2a (*P* < 0.05). The liver function indexes of both groups decreased gradually with the treatment time (*P* < 0.05) Figure 1.

### 3.4. Comparison of Marker Conversion

HBV-DNA, HBsAg, and HBeAg, which showed no evident difference between the two arms at T2 and T3 (*P* > 0.05), were lower in group 2b than in group 2a at T1 (*P* < 0.05). The quantitative detection results of HBV-DNA, HBsAg, and HBeAg in both groups showed a decreasing trend with the treatment time (*P* < 0.05). The two arms showed no evident difference in the negative conversion ratio of HBV-DNA, HBsAg, and HBeAg at T1, T2, and T3 (*P* > 0.05), as indicated by the statistical results of conversion (Figure 2 and Table 3).

### 3.5. Comparison of IFs

IL-1*β*, IL-6, IL-8, and TNF-*α*, which differed insignificantly between the two arms at T3 (*P* > 0.05), were lower in group 2b versus group 2a at T1 and T2 (*P* < 0.05). In both arms, these IFs decreased gradually with the treatment time (*P* < 0.05) Figure 3.

### 3.6. Comparison of Hemodynamics

SBP and DBP showed no distinct difference between the two arms at T1, T2, and T3 (*P* > 0.05); however, the MAP was higher and the CVP was lower in group 2b compared with group 2a (*P* < 0.05). During treatment, SBP and DBP of the two groups did not change significantly (*P* > 0.05), while MAP increased and CVP decreased gradually with the treatment time (*P* < 0.05) Figure 4.

### 3.7. Comparison of Cardiac Function

In the course of treatment, LVEF in both arms increased with the treatment time, while BNP decreased (*P* < 0.05). At T1, LVEF was significant higher in group 2b while the level of BNP was significant lower than in group 2a (*P* < 0.05) Figure 5.

### 3.8. Comparison of Treatment Safety

Comparison was also made on the incidence of ARs during treatment. The two arms had similar cases of fever, fatigue, insomnia, skin itching, and thyroid dysfunction (*P* > 0.05), while the cases with alopecia, thrombocytopenia, and granulocytopenia were fewer in group 2a compared with group 2b (*P* < 0.05) Table 4.

### 3.9. Comparison of Prognosis

During the 2-year follow-up, 40 patients in group 2a and 41 patients in group 2b were successfully followed up. The positive seroconversion rate of HBsAg and HBeAg differed insignificantly between the two arms (*P* > 0.05) Figure 6.

## 4. Discussion

CHB, as a highly contagious and occult disease, should be brought to the forefront of the clinic and patients [18]. Although there are stable and effective vaccines for CHB, there is still a certain periodicity in the existence of CHB vaccines in humans. Research indicates that people need to be vaccinated again 10-15 years after CHB vaccination to maintain the integrity of CHB antibodies [19]. However, most patients ignore the time of CHB vaccine revaccination, resulting in HBV infection in the process of antibody failure [20]. Therefore, reducing the threat of CHB lies in improving people's awareness of vaccination and preventing HBV infection on the one hand and in getting timely and effective clinical treatment on the other hand. PEG-IFN*α*-2a and PEG-IFN*α*-2b are currently the main clinical treatment options for CHB, and the merits and demerits of the two have always been an urgent issue to be verified in clinical research. This study, by comparing the efficacy of PEG-IFN*α*-2a and PEG-IFN*α*-2b in the treatment of HBeAg-positive CHB patients, is of important reference significance for future clinical selection of therapeutic drugs.

In this study, we first compared the clinical efficacy and found no difference in the overall response rate between the two arms, which suggested that both PEG-IFN*α*-2a and PEG-IFN*α*-2b had excellent therapeutic effects on CHB. Dogan et al. [12] compared the efficacy of pegylated interferon *α*-2a and *α*-2b in chronic hepatitis B patients and found that there were no significant differences between Peg-IFN*α*-2a and Peg-IFN*α*-2b treatment groups in achieving an SVR and undetectable HBV-DNA levels. Besides, the efficacy of PEG-IFN*α*-2a and PEG-IFN*α*-2b as the most commonly used drugs for treating CHB has been verified in many studies [21, 22], so the results obtained in this research are not out of expectation. Whereas, the merits and demerits of the two treatments need to be confirmed through various investigations. Furthermore, the liver function recovery was investigated. The results showed that after treatment, the indexes of liver function injury in both groups showed a decreasing trend, which further proved the therapeutic effect of both treatments on liver function. At T1, however, the reduction of ALT, AST, HA, LN, and IV-C was more significant in group 2b, suggesting that PEG-IFN*α*-2b could repair patients' liver function more quickly. At the same time, the detection results of CHB markers conversion showed that the negative conversion ratio of HBV-DNA, HBsAg, and HBeAg was consistent in the two groups after treatment; however, at T1, group 2b had lower HBV-DNA, HBsAg, and HBeAg as indicated by the quantitative test results with more patients showing complete response. As we all know, the key to the treatment of CHB lies in the inhibition of HBV-DNA polymerase activity [23]. HBsAg is the surface antigen of HBV-DNA particles, which can accelerate HBV maturation and complexity, while HBeAg is a soluble protein that can reflect HBV replication [24]. PEG-IFN*α*-2a and PEG-IFN*α*-2b are produced by combining polyethylene glycol molecules with a certain molecular weight on the basis of *α*-IFN, which can improve HBV-specific antibody levels in patients by enhancing oxidative metabolism, membrane depolarization, and phagocytosis [25].

Therefore, under the same pathway of action, we speculated that the reason for the difference between the two groups might be related to the molecular weight of the two kinds of IFN genes. PEG-IFN*α*-2a has a large molecular weight of about 40KD and better protection of IFN, so its blood concentration is more stable and its half-life is longer. However, due to its large molecular weight, PEG-IFN*α*-2a is mainly concentrated in blood and liver tissues after being injected into human body [26]. Because of this, some PEG-IFN*α*-2a drugs cannot be metabolized completely *in vivo* as the individual blood volume varies, so the liver function repair of some patients is slow in the initial use process. PEG-IFN*α*-2b, on the other hand, is only 12KD and has a wider distribution in the body. After injection, it can complete drug metabolism in blood, muscle, tissue, fat, and even cells [27], so it has a more rapid and significant effect on patients at the initial stage of use.

In addition, continuous HBV replication and the resulting immune-mediated response are important factors leading to hepatocyte inflammatory necrosis and hepatofibrosis. Excessive inflammatory reaction and fibrosis of hepatocytes will further destroy hepatocytes [28]. Therefore, in the treatment of CHB, anti-inflammatory effect is also one of the most important links. In this study, PEG-IFN*α*-2b showed faster inhibition of inflammation, which may also be related to our above inference. The occurrence of inflammatory reaction is a complicated pathological process, in which IFs are dominant, and cytokines such as monocytes and eosinophils are also involved [29]. As aforementioned, PEG-IFN*α*-2a works only in liver and blood and does not affect the activity cycle of cells, so its anti-inflammatory response is not as significant as PEG-IFN*α*-2b, an IFN gene involved in the cell life cycle. Similarly, the liver, as the most important metabolic organ in the human body, has a vital influence on the hemodynamics of the human body, and the most direct effect of hemodynamics is on the pumping capacity of the heart [30, 31]. While comparing the hemodynamic and cardiac functions of the two groups, we also found that PEG-IFN*α*-2b had a more significant improvement effect on MAP, CVP, LVEF, and BNP at the initial stage of treatment. This also verified our point of view again, indicating that PEG-IFN*α*-2b had a more comprehensive and rapid action in humans. However, a higher incidence of alopecia, thrombocytopenia, and granulocytopenia was identified in group 2b than in group 2a, suggesting a higher safety profile for PEG-IFN*α*-2a. It is also because PEG-IFN*α*-2a can be completely metabolized by the liver after the interference effect is completed, while PEG-IFN*α*-2b has a certain inhibitory effect on more cytokines, thus contributing to the reduction of such cells. It is also possible that PEG-IFN*α*-2b contains a higher number of IFN molecules (specific activity) per milligram of protein (PEG-IFN*α*-2b has a specific activity of 108 versus 107 of PEG-IFN*α*-2a) [32].

Finally, the follow-up results revealed no difference in the prognostic QOL and recurrence of CHB between the two arms, indicating that both treatments had stable long-term effect and high application value. However, through previous studies, we also found that the production rate of neutralizing antibodies against PEG-IFN*α*-2b was only about 3%, while that of PEG-IFN*α*-2a was about 6%-10% [33], which indicated that PEG-IFN*α*-2b was more effective in the long-term treatment of CHB. In our research, there was no difference in the prognosis between the two groups, which may be due to the small difference in the rate of neutralizing antibody production between the two groups on the one hand, or the chance caused by the short follow-up time or the small number of cases on the other hand.

However, the study still has some limitations, and due to the small base of research participants, we need to further expand the sample size to improve the comprehensiveness of experimental results. In addition, this paper proposed that the molecular weight difference between PEG-IFN*α*-2a and PEG-IFN*α*-2b was responsible for the differential performance of CHB treatment, which needs to be confirmed by further *in vitro* experiments, and the underlying mechanism needs to be clarified. In the future, we will conduct more in-depth and comprehensive experimental analysis on the treatment of CHB to obtain more effective experimental results for clinical reference.

## 5. Conclusion

Both PEG-IFN*α*-2a and PEG-IFN*α*-2b have excellent and stable therapeutic effects on HBeAg-positive CHB, among which PEG-IFN*α*-2b has a faster therapeutic process but higher side effects. These findings can provide reference for future clinical treatment of CHB.

## Figures and Tables

**Figure 1:** Comparison of liver function. (a) Comparison of ALT. (b) Comparison of AST. (c) Comparison of HA. (d) Comparison of LN. (e) Comparison of IV-C. Compared with 2b group, ^∗^*P* < 0.05. Compared with T1, ^#^*P* < 0.05. Compared with T2, ^&^*P* < 0.05.

**Figure 2:** Comparison of marker conversion. (a) Comparison of quantitative results of HBsAg. (b) Comparison of quantitative results of HBeAg. (c) Comparison of quantitative results of HBV-DNA. Compared with 2b group, ^∗^*P* < 0.05. Compared with T1, ^#^*P* < 0.05. Compared with T2, ^&^*P* < 0.05.

**Figure 3:** Comparison of inflammatory factors. (a) Comparison of IL-1*β* levels. (b) Comparison of IL-6 levels. (c) Comparison of IL-8 levels. (d) Comparison of TNF-*α* levels. Compared with 2b group, ^∗^*P* < 0.05. Compared with T1, ^#^*P* < 0.05. Compared with T2, ^&^*P* < 0.05.

**Figure 4:** Comparison of hemodynamics. (a) Comparison of SBP. (b) Comparison of DBP. (c) Comparison of MAP. (d) Comparison of CVP. Compared with 2b group, ^∗^*P* < 0.05. Compared with T1, ^#^*P* < 0.05. Compared with T2, ^&^*P* < 0.05.

**Figure 5:** Comparison of cardiac function. (a) Comparison of LVEF. (b) Comparison of BNP. Compared with 2b group, ^∗^*P* < 0.05. Compared with T1, ^#^*P* < 0.05. Compared with T2, ^&^*P* < 0.05.

**Figure 6:** Comparison of prognosis. (a) Comparison of social functioning scores. (b) Comparison of role-emotional scores. (c) Comparison of mental health scores. (d) Comparison of vitality scores. (e) Comparison of positive seroconversion rate of HBsAg. (f) Comparison of positive seroconversion rate of HBeAg.

**Table 1:** Comparison of clinical baseline data [*n*(%)].

	Group 2a (*n* = 42)	Group 2b (*n* = 42)	*t*/*χ*^2^	*P*
Age (years, ^−^*χ* ± *s*)	47.6 ± 8.2	46.4 ± 8.3	0.667	0.507
Gender [*n*(%)]			0.441	0.507
Male	23 (54.76)	26 (61.90)		
Female	19 (45.24)	16 (38.10)		
Family history of illness [*n*(%)]			0.124	0.724
Have	4 (9.52)	5 (11.90)		
Without	38 (90.48)	37 (88.10)		
History of liver disease [*n*(%)]			0.081	0.776
Have	8 (19.05)	7 (16.67)		
Without	34 (80.95)	35 (83.33)		
History of diabetes [*n*(%)]			0.223	0.637
Have	12 (28.57)	14 (33.33)		
Without	30 (71.43)	28 (66.67)		
History of hypertension [*n*(%)]			0.214	0.643
Have	15 (35.71)	13 (30.95)		
Without	27 (64.29)	29 (69.05)		
Smoking [*n*(%)]			0.449	0.503
Yes	18 (42.86)	15 (35.71)		
No	24 (57.14)	27 (64.29)		
Drinking [*n*(%)]			—	—
Yes	15 (35.71)	15 (35.71)		
No	27 (64.29)	27 (64.29)		
Living environment [*n*(%)]			0.343	0.558
City	34 (80.95)	36 (85.71)		
Countryside	8 (19.05)	6 (14.29)		

**Table 2:** Clinical efficacy [*n*(%)].

	Markedly effective	Effective	Invalid	Total effective rate (%)
Group 2a (*n* = 42)	21 (50.00)	14 (33.33)	7 (16.67)	83.33
Group 2b (*n* = 42)	24 (57.14)	14 (33.33)	4 (9.52)	90.48
*χ* ^2^				0.942
*P*				0.332

**Table 3:** Comparison of marker conversion [*n*(%)].

	Group 2a (*n* = 42)	Group 2b (*n* = 42)	*χ* ^2^	*P*
HBV-DNA negative conversion rate				
T1	8 (19.05)	13 (30.95)	1.587	0.208
T2	24 (57.14)	25 (59.52)	0.049	0.825
T3	34 (80.95)	36 (85.71)	0.343	0.558
HBsAg negative conversion rate				
T1	1 (2.38)	2 (4.76)	0.346	0.557
T2	3 (7.14)	4 (9.52)	0.156	0.693
T3	5 (11.90)	5 (11.90)	—	—
HBeAg negative conversion rate				
T1	8 (19.05)	10 (23.81)	0.283	0.595
T2	14 (33.33)	15 (35.71)	0.053	0.819
T3	22 (52.38)	24 (57.14)	0.192	0.661

**Table 4:** Incidence of adverse reactions [*n*(%)].

	Fever	Fatigue	Thyroid dysfunction	Alopecia	Insomnia	Skin itching	Thrombocytopenia	Granulocytopenia
Group 2a (*n* = 42)	14 (33.33)	19 (45.24)	4 (9.52)	6 (14.29)	10 (23.81)	1 (2.38)	11 (26.19)	24 (57.14)
Group 2b (*n* = 42)	15 (35.71)	21 (50.00)	5 (11.90)	15 (35.71)	11 (26.19)	1 (2.38)	20 (47.62)	33 (78.57)
*χ* ^2^	0.053	0.191	0.124	5.143	0.063	—	4.141	4.421
*P*	0.819	0.662	0.724	0.023	0.801	—	0.042	0.036

## Data Availability

The simulation experiment data used to support the findings of this study are available from the corresponding author upon request.
